This article has been retracted.

# Hyponatremia in Acute Stroke: A Comparative Study of Ischemic and Hemorrhagic Stroke Subtypes

**DOI:** 10.7759/cureus.91396

**Published:** 2025-09-01

**Authors:** Zahid Hasan, Murad Ali, Zia Ur-Rehman, Imran Qadar Khattak, Hamza Israr, Aansa Amin, Asim Ali, Amjad Ali

**Affiliations:** 1 Neurology, Mardan Medical Complex, Mardan, PAK; 2 Medicine, Bacha Khan Medical College, Mardan, PAK; 3 Pediatric Cardiology, Maqsood Medical Complex (MMC) General Hospital, Peshawar, PAK; 4 Internal Medicine, Hayatabad Medical Complex Peshawar, Peshawar, PAK; 5 General Internal Medicine, Mardan Medical Complex, Mardan, PAK

**Keywords:** acute confusion, acute stroke subtypes, cerebral edema, electrolyte imbalance, hemorrhagic stroke, hyponatremia, ischemic stroke

## Abstract

Background: Hyponatremia, an often underappreciated electrolyte imbalance in acute stroke, may exacerbate cerebral edema and negatively impact clinical outcomes. Although both ischemic and hemorrhagic strokes can be affected, there is a paucity of studies comparing the prevalence and severity of hyponatremia between these subtypes, particularly in resource-limited settings.

Objective: This study aims to ascertain the prevalence and severity of hyponatremia in patients with ischemic and hemorrhagic strokes and to compare subtype-specific differences in clinical and biochemical profiles.

Methods: This descriptive cross-sectional study involved 158 consecutive adult patients who presented with radiologically confirmed acute stroke within 24 hours of onset at a tertiary care hospital in Pakistan between December 2023 and March 2024. Patients were categorized into ischemic or hemorrhagic stroke subtypes based on computed tomography (CT)/magnetic resonance imaging (MRI) findings. Hyponatremia was considered a serum sodium concentration < 135 mmol/L, confirmed on two separate occasions 12 hours apart. Demographic, clinical, and biochemical data were collected. Statistical analyses included chi-square tests, t-tests, and multivariable logistic regression to adjust for confounders, with statistical significance set at p < 0.05.

Results: Hyponatremia was observed in 33% of patients, with a significantly higher prevalence in hemorrhagic stroke compared to ischemic stroke. Patients with hemorrhagic stroke had 5.2 times greater odds of hyponatremia. The distribution of hyponatremia severity was similar across stroke subtypes. Serum sodium levels were significantly lower in the hemorrhagic group. No significant associations were found between hyponatremia and age or sex.

Conclusion: Hyponatremia is significantly more prevalent in hemorrhagic stroke than in ischemic stroke, which indicates that close monitoring and early intervention are needed in these patients. Despite the similar severity distributions, the elevated risk in hemorrhagic stroke highlights the need for subtype-specific strategies in electrolyte management during acute stroke care.

## Introduction

Hyponatremia (serum sodium < 135 mmol/L), a prevalent yet underappreciated electrolyte abnormality [1], frequently afflicts patients with acute stroke, impacting 15%-50% of this population [2]. This electrolyte imbalance can exacerbate cerebral edema, prolong hospitalizations, and increase mortality rates, thereby contributing to poorer outcomes [3]. While stroke remains a leading cause of global disability, with ischemic stroke comprising 85% of cases and intracerebral hemorrhage (ICH) associated with disproportionately high mortality [4], the subtype-specific burden and clinical implications of hyponatremia in acute stroke remain inadequately characterized [5]. This lack of understanding underscores the necessity for further investigation into the prevalence, severity, and impact of hyponatremia across different stroke subtypes.

Existing studies have significant limitations that hinder a comprehensive understanding of hyponatremia in acute stroke. First, most investigations have focused on a single stroke subtype, either ischemic [6] or hemorrhagic [7], without directly comparing the two. This subtype-specific approach fails to capture the potential differences in the prevalence and implications of hyponatremia between ischemic and hemorrhagic stroke. Second, large database analyses often lack detailed clinical data, while single-center studies from high-income settings may not be generalizable to resource-limited regions.

The aim of this cross-sectional study is to determine the prevalence and severity of hyponatremia in patients with ischemic and intracerebral hemorrhagic stroke. It also seeks to compare the severity of hyponatremia between these two stroke subtypes while accounting for potential confounding factors. Understanding the distribution of severity is important, as greater hyponatremia severity has been associated with worse neurological outcomes, longer hospital stays, and higher complication rates [8]. By identifying these patterns, this study intends to inform targeted electrolyte monitoring strategies, thereby helping to prevent and reduce preventable complications in patients suffering from acute stroke.

## Materials and methods

This descriptive cross-sectional study was conducted at the Medical A Ward of Mardan Medical Complex, a tertiary care hospital in Khyber Pakhtunkhwa, Pakistan, from December 2023 to March 2024. The study protocol received approval from the Institutional Review Board of Bacha Khan Medical College, Mardan (approval number 435).

All adult patients presenting with acute stroke meeting the following inclusion and exclusion criteria and presenting within 24 hours of symptom onset were enrolled using a non-probability consecutive sampling technique. Inclusion criteria comprised radiologically confirmed acute ischemic stroke (AIS), indicated by a hypodense lesion on non-contrast computed tomography (CT) brain or a hyperintense lesion on diffusion-weighted magnetic resonance imaging (MRI), and primary intracerebral hemorrhage, identified by spontaneous intraparenchymal hemorrhage on CT scan. Exclusion criteria included secondary intracranial conditions, comorbidities predisposing to hyponatremia, and current use of diuretics or other medications affecting sodium homeostasis.

The minimum sample size was estimated using the World Health Organization (WHO) Sample Size Calculator based on an expected prevalence of hyponatremia in acute stroke of 11.6% (95% confidence interval (CI), 5% margin of error, and design effect of 1.0). After data collection, a post hoc power analysis (two-proportion comparison, two-sided α = 0.05) using the observed prevalences (21.6% (24/111) (AIS) versus 59.6% (28/47) (ICH)) and group sizes (n = 111 and n = 47) demonstrated achieved power = 0.996, confirming adequacy to detect the observed difference. A sensitivity analysis indicated that, with the same sample sizes, an ICH prevalence of approximately 44% (versus AIS prevalence of 21.6%) would provide ≥80% power.

Data collection included a clinical assessment involving baseline demographic and medical history recording, a neurological examination with National Institutes of Health (NIH) Stroke Scale scoring [9], laboratory investigations such as serum electrolyte measurement via ion-selective electrode, renal, liver, and thyroid function evaluation, full blood count, and neuroimaging consisting of non-contrast computed tomography brain scans for all participants and magnetic resonance imaging brain scans when clinically indicated. Hyponatremia was defined as a serum sodium concentration below 135 mmol/L, confirmed on two separate occasions, at least 12 hours apart [10]. Stroke subtypes were classified as acute ischemic stroke, characterized by acute neurological deficit with corresponding CT or MRI findings, and intracerebral hemorrhage, defined as spontaneous intraparenchymal bleeding without associated trauma.

Statistical analyses were performed using IBM SPSS Statistics software version 24.0 (IBM Corp., Armonk, NY). Continuous variables were summarized as mean ± standard deviation (SD). Distributions were visually inspected using histograms and boxplots, which suggested approximate symmetry; therefore, formal normality tests (e.g., Shapiro-Wilk) and homogeneity of variance (e.g., Levene's test) were not applied. This approach allowed for consistent reporting of central tendency and variability across all variables. Categorical variables were summarized using frequencies and percentages. Group comparisons involved chi-square or Fisher's exact test for categorical variables, and independent samples t-tests for continuous variables.

Binary logistic regression was employed to evaluate the association between stroke subtype (ischemic versus hemorrhagic) and hyponatremia, while adjusting for potential confounding variables (e.g., age, sex, hypertension, diabetes, and comorbidities). Odds ratios (ORs) with corresponding 95% confidence intervals (CIs) were reported to quantify the strength and precision of associations. Statistical significance was set at p < 0.05. Formal model fit statistics (e.g., Hosmer-Lemeshow test) and multicollinearity diagnostics (e.g., variance inflation factor (VIF)) were not performed, which represents a limitation of the study.

Written informed consent was obtained from all participants or their legally authorized representatives, ensuring patient confidentiality through anonymized data collection and secure storage.

## Results

The study cohort consisted of 158 patients diagnosed with acute stroke. The mean age of the cohort was 60.0 ± 2.7 years, with men comprising 62% of the study population. The mean age was significantly higher in patients with hemorrhagic stroke (61.8 ± 3.1 years) compared to those with ischemic stroke (59.2 ± 2.5 years), and this difference was statistically significant (t = -5.09, p < 0.001). In contrast, the distributions of sex between the two stroke subtypes were not significantly different between the ischemic and hemorrhagic stroke subtypes (χ² = 0.00, p = 1.000), as shown in Table 1*.*

**Table 1:** Baseline Characteristics by Stroke Type Data presented as numbers (%) or mean ± SD. Key: Chi-square test was used for categorical variables, and the independent samples t-test was used for continuous variables. A p-value < 0.05 was considered significant; a p-value < 0.001 was considered highly significant. SD: standard deviation

Variable	Total (N = 158)	Ischemic (n = 111)	Hemorrhagic (n = 47)	Test statistics	p-value
Age, mean ± SD	60.0 ± 2.7	59.2 ± 2.5	61.8 ± 3.1	t = -5.09	<0.001
Male sex, number (%)	98 (62%)	69 (62.2%)	29 (61.7%)	χ² = 0.00	1.000

Hyponatremia was observed in 33% of the total patient population. The incidence of hyponatremia was notably higher in hemorrhagic stroke compared to ischemic stroke. Logistic regression analysis indicated that patients with hemorrhagic stroke had significantly higher odds of developing hyponatremia compared to patients with ischemic stroke, with an odds ratio of 5.2 (95% CI: 2.9-8.8, p < 0.001) (Table 2)*.*

**Table 2:** Hyponatremia Prevalence by Stroke Type Data are presented as numbers (%). Logistic regression analysis was used to calculate the OR for associations. A p-value < 0.05 was considered statistically significant. OR: odds ratios

Stroke type	With hyponatremia	Without hyponatremia	OR	p-value
Ischemic (n = 111)	24 (21.6%)	87 (78.4%)	Reference	<0.001
Hemorrhagic (n = 47)	28 (59.6%)	19 (40.4%)	5.2	

Stratified analysis by demographics revealed no significant difference in the prevalence of hyponatremia between the age groups of 30-50 years and 51-70 years. Similarly, the prevalence of hyponatremia was found to be comparable between male and female patients. 

The severity of hyponatremia was comparably distributed between patients with ischemic and hemorrhagic stroke. Among patients with ischemic stroke, 15 cases had mild, seven had moderate, and two had severe hyponatremia. Likewise, in patients with hemorrhagic stroke, 18 cases were mild, eight were moderate, and two were severe. There was no statistically significant difference in the severity distribution between the two stroke subtypes (all: p > 0.89), indicating that while the overall prevalence of hyponatremia was higher in patients with hemorrhagic stroke, the degree of severity remained similar across the groups (Table 3)*.*

**Table 3:** Hyponatremia Severity Distribution Data are presented as frequencies. This table includes only patients with hyponatremia. For total counts per group (with/without hyponatremia), refer to Table 2. Statistical significance was assessed using Fisher's exact test to compare the distribution of hyponatremia severity between ischemic and hemorrhagic stroke types. A p-value < 0.05 was considered statistically significant.

Severity	Ischemic (n = 24) (number (%))	Hemorrhagic (n = 28) (number (%))	Fisher's exact	p-value
Mild	15 (62.5%)	18 (64.3%)	0.893	0.893
Moderate	7 (29.2%)	8 (28.6%)	1.000	1.000
Severe	2 (8.3%)	2 (7.1%)	1.000	1.000

In summary, the incidence of hyponatremia was significantly higher among patients with hemorrhagic stroke, with these patients exhibiting 5.2 times greater odds (95% CI: 2.9-8.8) of developing hyponatremia compared to those with ischemic stroke. However, no significant differences were observed in the distribution of hyponatremia severity or its association with age or sex. These findings underscore the importance of closely monitoring serum sodium levels, particularly in patients presenting with hemorrhagic stroke.

## Discussion

This study emphasizes the considerable prevalence of hyponatremia in acute stroke patients, highlighting the necessity of consistent electrolyte monitoring in stroke management. The results indicate a notable difference in hyponatremia prevalence between stroke subtypes, with 60% of patients with hemorrhagic stroke affected, compared to 22% of patients with ischemic stroke. Although hemorrhagic stroke showed a significantly higher incidence of hyponatremia, the 22% prevalence in ischemic stroke remains clinically relevant, affecting nearly one-quarter of these patients. Severity stratification revealed similar distributions across subtypes, suggesting comparable pathophysiological patterns once hyponatremia develops. The study's findings suggest that while hyponatremia is observed in both ischemic and hemorrhagic stroke subtypes, its occurrence is significantly higher in hemorrhagic stroke, with a 5.2-fold increased likelihood compared to ischemic stroke. These results underscore the potential impact of sodium imbalance on stroke outcomes and emphasize the importance of implementing tailored management approaches for these patients.

These findings align with existing literature, which reports varying rates of hyponatremia in patients with stroke. Prior research indicates a prevalence range of 15%-25% in ischemic stroke and 40%-60% in hemorrhagic stroke [11]. The higher prevalence observed in patients with hemorrhagic stroke is consistent with evidence suggesting a greater predisposition to cerebral salt wasting (CSW) and syndrome of inappropriate antidiuretic hormone secretion in this subtype [12,13]. However, the direct comparison of these stroke subtypes within a single cohort renders this study a noteworthy contribution to the existing literature.

Our results support the work of Rafat et al., who highlighted that even mild hyponatremia in ischemic stroke patients is associated with increased cerebral edema and poorer neurological outcomes [14]. The implications are even more significant for hemorrhagic stroke, as sodium imbalances can exacerbate osmotic shifts, potentially leading to secondary brain injury. Given the substantially higher likelihood of hyponatremia in patients with hemorrhagic stroke, early identification and management of sodium disturbances should be prioritized.

The differential diagnosis of hyponatremia in patients with stroke includes syndromes of inappropriate antidiuretic hormone (SIADH) and cerebral salt wasting (CSW), each requiring distinct treatment approaches. The manifestation of these disorders can differ by stroke type. SIADH is a common response to brain injury in both ischemic and hemorrhagic strokes. CSW, however, is more predominantly linked to hemorrhagic strokes, particularly subarachnoid hemorrhage, where cerebral irritation and elevated natriuretic peptides drive renal salt excretion; it is seen less frequently in large-volume ischemic strokes that significantly increase intracranial pressure or affect central autonomic centers [13].

For patients with ischemic stroke, hyponatremia management should focus on identifying and treating underlying causes, such as SIADH or volume depletion, to prevent worsening neurological outcomes. Conversely, for patients with hemorrhagic stroke, where hyponatremia prevalence is significantly higher, aggressive sodium correction and close monitoring should be considered to mitigate the risk of secondary brain injury resulting from osmotic imbalances.

The strength of this study is in its comparative analysis of hyponatremia prevalence between ischemic and hemorrhagic stroke subtypes within a South Asian population, providing valuable regional insights. Furthermore, the use of standardized sodium measurement methods and strict exclusion criteria enhances the reliability of the results.

Considering the clinical significance of the present study's findings, future research should focus on several important areas. Multicenter validation studies are needed to corroborate the observed prevalence rates across various populations. Further mechanistic research on the specific roles of SIADH versus cerebral salt wasting in patients with stroke with hyponatremia would help clarify the underlying pathophysiology. Lastly, interventional studies to assess the effects of specific sodium management approaches on stroke recovery and long-term outcomes would greatly benefit the existing literature.

Several limitations should be considered when interpreting this study. First, its single-center setting may restrict the generalizability of the findings to other settings and populations. Second, the absence of urinary electrolyte data prevents differentiation between syndrome of inappropriate antidiuretic hormone and cerebral salt wasting, thereby limiting the interpretation of underlying mechanisms. Third, the short follow-up period did not allow for assessing long-term functional outcomes related to hyponatremia, which could have provided valuable insights into patient prognosis. Finally, certain methodological limitations should be acknowledged: formal statistical testing for normality (e.g., Shapiro-Wilk test) was not performed, with distributions instead assessed visually and summarized as mean ± SD, which may limit the precision of distributional assumptions. In addition, regression diagnostics, such as the Hosmer-Lemeshow test for model fit and variance inflation factors (VIFs) for multicollinearity, were not conducted. Although odds ratios with 95% confidence intervals were reported, the absence of these diagnostic checks may restrict the robustness and interpretability of the regression findings.

## Conclusions

In conclusion, this study demonstrates that hyponatremia is significantly more prevalent among patients with hemorrhagic stroke compared to those with ischemic stroke, with a 5.2-fold higher risk identified in the former group. This disparity is not merely of statistical importance but carries substantial clinical implications. Hyponatremia has been consistently associated with adverse neurological outcomes, including exacerbation of cerebral edema, heightened risk of seizures, prolonged hospitalization, and increased morbidity and mortality. The disproportionate burden observed in hemorrhagic stroke therefore underscores the necessity of incorporating vigilant sodium monitoring and proactive management into standard care protocols for these patients. Although the severity distribution of hyponatremia did not differ significantly between stroke subtypes, its higher prevalence in hemorrhagic stroke highlights the importance of routine electrolyte assessment as an integral component of acute stroke care. Early detection and tailored therapeutic strategies may mitigate neurological deterioration, prevent secondary complications, and optimize short-term outcomes. Future research should focus on delineating the underlying pathophysiological mechanisms driving this association while also exploring the long-term prognostic implications of hyponatremia in both ischemic and hemorrhagic stroke through multicenter, longitudinal studies. Such evidence would be pivotal in guiding more precise management algorithms and improving the overall quality of stroke care.

## References

[1] Khan A, Khan Z, Khan S, Ullah A, Ayub G, Tariq MN (2023). Frequency of hyponatremia and its impact on prognosis in ischemic stroke. Cureus.

[2] Barkas F, Anastasiou G, Liamis G, Milionis H (2023). A step-by-step guide for the diagnosis and management of hyponatraemia in patients with stroke. Ther Adv Endocrinol Metab.

[3] Yuen KC, Sharf V, Smith E, Kim M, Yuen AS, MacDonald PR (2022). Sodium and water perturbations in patients who had an acute stroke: clinical relevance and management strategies for the neurologist. Stroke Vasc Neurol.

[4] Flynn RW, MacWalter RS, Doney AS (2008). The cost of cerebral ischaemia. Neuropharmacology.

[5] Rodrigues B, Staff I, Fortunato G, McCullough LD (2014). Hyponatremia in the prognosis of acute ischemic stroke. J Stroke Cerebrovasc Dis.

[6] Mahesar SA, Memon SF, Mustafa S, Javed A, Butt SM (2019). Evaluation of hyponatremia in ischemic stroke patients in a tertiary care hospital of Karachi, Pakistan. Cureus.

[7] Kuramatsu JB, Bobinger T, Volbers B (2014). Hyponatremia is an independent predictor of in-hospital mortality in spontaneous intracerebral hemorrhage. Stroke.

[8] Zafar M, Jalil A, Ghaffer A, Yousaf M, Batool S (2024). Hyponatremia in ischemic stroke patients and its relationship to clinical outcomes in such patients. J Rawalpindi Med Coll.

[9] Thomas SE, Plumber N, Venkatapathappa P, Gorantla V (2021). A review of risk factors and predictors for hemorrhagic transformation in patients with acute ischemic stroke. Int J Vasc Med.

[10] Adrogué HJ, Tucker BM, Madias NE (2022). Diagnosis and management of hyponatremia: a review. JAMA.

[11] Hossain MF, Kharel M, Husna AU, Khan MA, Aziz SN, Taznin T (2023). Prevalence of electrolyte imbalance in patients with acute stroke: a systematic review. Cureus.

[12] Cui H, He G, Yang S, Lv Y, Jiang Z, Gang X, Wang G (2019). Inappropriate antidiuretic hormone secretion and cerebral salt-wasting syndromes in neurological patients. Front Neurosci.

[13] Shah A, Sabir S, Artani M, Salam O, Khan S, Rizwan A (2019). Significance of hyponatremia as an independent factor in predicting short-term mortality in patients with hemorrhagic stroke. Cureus.

[14] Rafat C, Flamant M, Gaudry S, Vidal-Petiot E, Ricard JD, Dreyfuss D (2015). Hyponatremia in the intensive care unit: how to avoid a Zugzwang situation?. Ann Intensive Care.

